This article has been retracted.

# Positioning of Prefabricated Building Components Based on BIM and Laser Image Scanning Technology in the Environment of Internet of Things

**DOI:** 10.1155/2022/5976935

**Published:** 2022-06-23

**Authors:** Yuting Zhong, Zesheng Qin

**Affiliations:** Department of Civil Engineering, Southeast University, Nanjing 211189, Jiangsu, China

## Abstract

In order to accurately locate the fabricated building components during assembly, the fabricated building components are monitored by laser scanning. At the same time, BIM Technology is proposed to carry out construction management in the construction process, realize safe site management and construction, reduce unnecessary mistakes of human operation, and improve construction quality. With the progress of computer technology, the emergence of the Internet of things has brought convenience to many fields. This research uses the application of phase ranging to carry out omnidirectional laser scanning on the fabricated building components, obtain the point cloud data, and use BIM Technology to simulate and analyze the building, establish the accurate positioning of building components, and prevent the offset phenomenon in the assembly process, so as to improve the construction quality and efficiency. In recent years, the integration of information technology into prefabricated buildings plays a vital role in the transformation and upgrading of China's construction industry. At the same time, it will also raise the information management level of prefabricated buildings to a new level. In order to improve the quality of building construction, this paper proposes a positioning method of prefabricated building components based on BIM Technology and laser scanning. On this basis, a complete architecture and detailed process application are established, and the promotion policies conducive to the development of intelligent construction of prefabricated buildings in BIM are put forward.

## 1. Introduction

China's population base enlarges the demand for housing and promotes the rapid development of technology in the field of construction. In the past two decades, China has invested a lot of human and material resources in infrastructure construction, which has accelerated the process of urbanization. At the same time, the requirements for the construction field are constantly improving, which also stimulates the competition and innovation among the construction industry and improves the innovative technology in the construction field. In order to save production costs and reduce costs, prefabricated buildings have emerged [1].

Prefabricated buildings are standardized and customized from the source of design and mass-produced standard building components for unified allocation, installation, and management, so as to realize energy-saving and double carbon sustainable development of building component products [3]. The three-dimensional space technology can accurately locate the spatial information data, which is usually used in surveying and mapping, exploration, construction, high-altitude operation, and other aspects. The ground measuring instrument is used to locate the objects to be measured by laser scanning technology. In essence, it is to obtain a large number of three-dimensional coordinates of ranging points by measuring the distance by laser and integrate these data through calculation methods to obtain high-precision data information.

The survey work of Su et al. in infrastructure construction is more important. The traditional level cannot accurately obtain data, which increases the difficulty of follow-up work. In order to obtain the accurate data of the main beam alignment, the bridge alignment is measured by using three-dimensional laser scanning imaging technology, which can reduce the error in the measurement and improve the work efficiency [4]. Tan et al. reported a high production accuracy of aircraft spare parts, so using laser scanning imaging technology to detect spare parts can help alleviate the error caused by automatic production, improve the measurement accuracy, and promote the application of value in industrial production [5].

Three-dimensional laser scanning technology can obtain a large number of data coordinate points of the target and can accurately and quickly convert the data into three-dimensional data, so as to reduce the error of human operation and improve the accuracy and work efficiency.

In the past two decades, China's infrastructure has developed rapidly. With the continuous improvement of China's economic level, the population structure is also undergoing great changes. The promotion of urbanization has made the construction industry the industry that benefits the most from the demographic dividend. The application of BIM Technology in architectural design can use the relevant data of construction engineering to build simulation and improve the unity, relevance, coordination, and visualization of information, so as to improve the construction quality [6].

With the application of computer technology and BIM Technology in various fields, the requirements of visualization technology in various fields are higher and higher. This research mainly discusses the application of three-dimensional laser scanning technology combined with BIM Technology in prefabricated building components, so as to achieve accurate positioning between building components in the environment of Internet of things, so as to improve work efficiency.

## 2. Application of BIM Technology in Construction Engineering

Construction enterprises encounter some management conflicts in the process of project construction. In order to seek a reasonable development mode and strengthen the construction process management in combination with the enterprise's own situation, BIM Technology has become an effective measure to solve these conflicts in project construction management [3].

BIM has the following characteristics:

1. Optimized design and construction management: in some complex construction projects, due to the complex spatial layout and the intersection of various systems, the requirements for the layout of equipment pipelines and lines are high, and the conflict between equipment pipelines and lines is easy to occur, which brings some trouble to the construction process [7]. If you do not pay attention in the management, you will make mistakes, resulting in rework or repeated labor, increasing the cost in the construction process and delaying the construction period. At the same time, in the construction process of the main building, optimizing the construction scheme through software can avoid the defects in the theoretical design in the construction drawings, reasonably plan the construction sequence of the project, reduce the change of projects in the construction, and reduce unnecessary waste. BIM Technology can draw and summarize the professional models of architecture, structure, and fluid mechanics, sort out and import the relevant data into the software according to the needs of each discipline, and finally give a reasonable construction layout of pipeline, line, and structure, so as to realize overall management and reduce repeated work procedures in construction.
2. Interdisciplinary coordination: the construction process of construction projects will encounter the division of labor and cooperation among various professionals. Coordinating the mutual cooperation of various professionals in construction is an important process in project management. In order to ensure the smooth progress of construction, all professionals need to cooperate with each other to achieve the goal [8]. The project construction site needs professionals in civil engineering, HVAC, pipeline, fire protection, water, and electricity. Due to the influence of professional and technical differences, there is a lack of necessary communication and coordination between them, which often leads to local and potentially unforeseen problems, resulting in secondary rework during cross operation. BIM Technology can optimize such problems, simulate the construction process through visual and intelligent means, indicate the problems that may cause conflicts in advance, and coordinate various professionals to reduce technical errors and errors in the construction process.
3. Site layout optimization: the project construction site management is not only the management of the construction team, but also the reasonable layout of the complex environment around the project. Due to the different environment of the project construction site and the city's demand for civilized construction on the construction site, it is easy to bring some difficulties to the layout of the construction site. BIM Technology establishes the construction site model through relevant data, restores the real surrounding environment of the construction site, helps to simulate the site conditions at relevant stages, and effectively makes a reasonable layout of the construction site.
4. Quality management of construction site: in the process of project construction, errors occur frequently due to complex processes and large differences in the quality of personnel involved [9]. If necessary, rework and secondary management can be carried out in time, and the labor cost can be reduced. Through the comparison between BIM model and construction results, problems can be found in time and effectively, and problems can be intervened in time. The traditional on-site quality inspection personnel usually cannot achieve the accuracy of artificial intelligence, and the comparison of a large amount of data requires drawings and technical support, which requires a lot of manpower, which brings a lot of inconvenience to the construction site management. The application of BIM Technology can compare the construction information through the model and optimize and verify the quality problems.
5. Safety management: there are usually safety management personnel at the construction site to screen and publicize potential safety hazards, which often rely on the experience accumulated in long-term work [10]. BIM Technology in safety management can screen potential safety hazards by simulating the real environment of the site, give advance warning to the hazard sources in advance, find out the areas with hidden safety risks, restore the site risk factors through simulation, analyze the causes of accidents, and put forward corresponding rectification measures to prevent hazards and avoid personal injury.

## 3. Positioning Technology of Prefabricated Building Components

### 3.1. Positioning of Fabricated Building Components by Laser Image Scanning Technology

Prefabricated building is a building mode that has attracted more attention at present, especially in the process of urbanization construction, and the national policy encourages the promotion of prefabricated building [11]. The modular materials made of unified design, production, and processing are used to stack the components of the building. It is not suitable for buildings with too high floors, generally no more than the sixth floor, and there are certain requirements for material strength. Because modular materials can be processed in advance according to the building shape, it can save schedule time and cost for subsequent construction and reduce material waste and has a high degree of industrialization and certain flexibility. Mechanical assistance is required in the stacking process, which has strong operability and reduces labor intensity and personnel cost.

The modular parts of the building, such as interior and exterior wall modules, precast beam modules, air-conditioning panels, and other components, need to be accurately positioned during combination. The auxiliary machinery is used to splice the assemblies under manual operation. If the auxiliary machinery is operated manually to splice the components, a little carelessness will cause component damage and deformation, resulting in construction quality problems, material waste, manual repeated labor, and other problems. Three-dimensional laser scanning plays a monitoring role in the construction process. It can accurately locate the assemblies, realize the effective splicing between the assemblies, and reduce the risks brought by human operation errors to the construction process. The specific monitoring path is shown in Figure 1.

In Figure 1, the monitoring system plays an important role in the installation of building components. The 3D laser probe is arranged in all aspects to scan the components to be combined, and the auxiliary positioning information of the objects to be positioned in the air is used to form the 3D point cloud data. The relevant mapping relationship between the internal elements of the camera and the 2D image is established in the 3D space. Through the mapping relationship between 2D and 3D, so as to determine the three-dimensional point orientation between the targets, the obtained data are denoised by wavelet, the external interference is removed, and then the relevant data are obtained by neurofuzzy calculation, and the binary output calculation results are used. This process can make the model have more accurate spatial and geographical accuracy of monitoring and avoid errors in the process of combination.

### 3.2. Statistical Methods

In the research on the positioning method of assembled building components based on BIM Technology and laser image scanning technology, the calculation of machine learning fuzzy neural network needs a variety of data calculation methods. Firstly, the wavelet basis function is used to denoise various interference factors, and the wavelet basis function is shown in the following formula:

(1) $$\begin{array}{c} X\left(a,b\right)=\frac{1}{\sqrt{b}}\int_{-\infty }^{\infty }x\left(t\right)\psi \left(\frac{t-a}{b}\right)\text{d}t. \end{array}$$

As can be seen from the above formula, *ω* system frequency is a variable. Different variables from Fourier transform have only frequency, and wavelet function analysis has two variables: scale a and translation. Scale a controls the expansion and contraction of the wavelet function, and the scale is inversely proportional to the frequency *τ*. It corresponds to time.

If the fuzzy neural network is used to control the recent change law of time series data, or the minimum number of nodes is needed to realize the fuzzy convolution of data, the sixth-order polynomial depth Iterative Regression basis function with complex function curve and rich regression coefficients needs to be used, and its expression is shown in the following formula:

(2) $$\begin{array}{c} y=\overset{n}{\underset{i=1}{\sum }}\overset{5}{\underset{j=0}{\sum }}A_{j}x_{i}^{j}. \end{array}$$

Among them, *A*_*j*_ is the coefficient to be regressed of the *j*-th order polynomial; that is, each node in the formula contains 6 coefficients to be regressed from A0 to A5. *jis* is the polynomial order. The meanings of other mathematical symbols are the same as those above.

The node basis function of the binary neural network is shown in the following formula:

(3) $$\begin{array}{c} y=\overset{n}{\underset{i=1}{\sum }}\frac{1}{A+B\cdot e^{x_{i}}}. \end{array}$$

Among them, *e* is the natural constant; here, take the approximate value *E* = 2.718281828. The meaning of other mathematical symbols is the same as formulas (1) and (2) above.

## 4. Results

### 4.1. Comparison Results of R2 Fitting Curves Located in Different Ways

Python software is used to fit the straight curve of the test data. The result of curve fitting uses the value of R2 to judge the consistency between the data to be evaluated and the fitting function. The positioning data of intelligent positioning group and manual group in the rising section, translation section, and falling section are collected for curve fitting, and the data in Table 1 is obtained.

In Table 1, in the rising section, the *R*^2^ value of the intelligent positioning group is 0.974, while the R2 value of the manual group is only 0.756. In the translation section, the *R*^2^ value of the intelligent positioning group is 0.984, while the *R*^2^ value of the manual group is only 0.863. In the descending section, the *R*^2^ value of the intelligent positioning group is 0.915, while the *R*^2^ value of the manual group is only 0.733. From the comparison results of the *R*^2^ values of the two groups, it can be seen that the *R*^2^ value of the intelligent positioning group is much higher than that of the manual group. According to the *R*^2^ value data in the above table, as shown in Figure 2, the data difference between intelligent positioning group and manual group can be seen more clearly.

In Figure 2, it can be seen that the *R*^2^ value of the intelligent positioning group is closer to 1 than that of the manual group in the rising section, translation section, and falling section, which shows that the curve fitting results of the intelligent positioning group in the installation and positioning of building components have high consistency. The closer the *R*^2^ value is to 1, the higher the consistency is between the test data and the fitting function, which indicates that the moving track of the intelligent positioning group has a higher overlap with the ideal track.

### 4.2. Comparison Results of Work Efficiency between Intelligent Positioning Group and Manual Group

In order to verify the working efficiency of the prefabricated building component positioning based on BIM and laser image scanning technology in the practical application, the lifting efficiency and moving speed of the intelligent positioning group and the manual group are collected and analyzed to obtain the data in Table 2.

In Table 2, the hoisting efficiency of artificial intelligence group is 0.934, while that of artificial group is 0.621. The data comparison difference between the two groups has not only a certain threshold difference, but also statistical significance. The comparison results of the moving speeds of the two groups, whether the maximum speed, the minimum speed, or the average speed, show that the intelligent positioning group is higher than the manual group, so the work efficiency must be higher than that of the intelligent positioning group. See Figure 3 according to the data in Table 2 above.

In Figure 3, the data comparison results of the intelligent positioning group and the manual group in the lifting efficiency and lifting movement speed found that the indicators of the intelligent positioning group are better than those of the manual group, which also shows that the intelligent positioning group can locate the fabricated building components more accurately after using BIM and laser image scanning technology, thus indirectly improving the moving speed and lifting efficiency.

### 4.3. Comparison Results of Intelligent Positioning, Manual Rework, and Damage to Equipment

The rework, regular circulation, and damage of equipment of building construction installed in different ways are investigated by questionnaire, and then the results are analyzed to obtain the data in Table 3 below.

In Table 3, the data difference between the intelligent positioning group and the artificial group not only has a certain threshold difference but also has obvious statistical significance (*P* < 0.01). Moreover, the rework rate, regular circulation rate, and equipment damage rate of the intelligent positioning group are 1.96%, 96.72%, and 0.73%, respectively. The rework rate, regular circulation rate, and equipment damage rate of the manual group were 8.63%, 83.25%, and 3.65%, respectively. From the data, we can see that the rework rate and equipment damage rate of intelligent positioning group are lower than those of manual group, and the normal circulation rate of intelligent positioning group is higher than that of manual group. According to the data in the above table, see the following Figure 4.

In Figure 4, from the comparison of rework rate and damage rate of equipment, it can be seen that the rework rate of intelligent positioning group is much lower than that of equipment, which can also indirectly show that the application of intelligent positioning of prefabricated building components through BIM and laser image scanning technology can reduce the rework and damage of equipment, which can be widely used, which can improve the assembly efficiency of workers and save costs.

### 4.4. Comparison of Satisfaction Survey Results of Different Groups

In order to compare the advantages and disadvantages of the hoisting of prefabricated building components positioned by BIM and laser image scanning technology and manual hoisting, the satisfaction of participating merchants, operators, and customers was investigated, and the data in Table 4 below were obtained.

In Table 4, from the comparison of the satisfaction data of the two groups, it can be seen that the satisfaction of businesses, operators, and customers with the hoisting of prefabricated building components with intelligent positioning is better than that of the manual group. This also shows that the intelligent positioning method using BIM and laser image scanning technology is more popular.

In Figure 5, for the two groups of satisfaction data image comparison results, it can be seen that businesses, operators, and customers are relatively satisfied with the assembly mode of intelligent positioning building components, which also shows that the application of technology can help improve their work efficiency and quality of life.

## 5. Conclusion

In order to ensure the quality and safety management of fabricated building components in the construction process, the on-site environment is truly simulated through BIM Technology, and the process steps are optimized. With the progress of science and technology, the emergence of the Internet of things makes visualization further [12]. This research uses laser scanning imaging technology to scan the fabricated building components, which can effectively obtain the space real-time distance, help to accurately judge the assembled building components in combination, avoid manual operation errors and other potential safety hazards, improve the construction quality and efficiency, and reduce the secondary rework phenomenon and labor cost waste in the construction process. Artificial intelligence is fast and efficient with zero error, which brings revolutionary changes to industry and production and also brings convenience to the construction industry. We believe that the future world of artificial intelligence will be higher and lead the more efficient and accurate development of the construction industry.

## Figures and Tables

**Figure 1:** Monitoring path of laser image scanning technology in fabricated building components.

**Figure 2:** Comparative analysis of *R*^2^ values in different groups.

**Figure 3:** Comparison of work efficiency of different groups.

**Figure 4:** Comparison of equipment damage and rework.

**Figure 5:** Comparison of satisfaction between intelligent positioning group and manual group.

**Table 1:** *R* ^2^ value data results of intelligent positioning group and manual group.

Group	Rising section	Translation segment	Descending section
Artificial group	0.756	0.863	0.733
Intelligent positioning group	0.974	0.984	0.915
*t*	2.331	3.057	1.984
*P*	0.004	0.002	0.003

**Table 2:** Lifting efficiency and moving speed results of different groups.

Group	Hoisting efficiency (u/min)	Moving rate (m/s)		
		Maximum	Minimum	Average
Artificial group	0.621	2.25	0.17	1.08
Intelligent positioning group	0.934	2.84	0.93	1.46
*t*	1.267	8.029	2.284	3.691
*P*	0.008	0.006	0.007	0.006

**Table 3:** Comparison of rework and equipment damage under different positioning modes.

Group	Average rework rate (%)	Normal circulation rate (%)	Equipment damage rate (‰)
Artificial group	8.63	83.25	3.65
Intelligent positioning group	1.96	96.72	0.73
*t*	0.000	1.566	0.000
*P*	0.003	0.002	0.004

**Table 4:** Satisfaction of different assembly methods.

Group	Business satisfaction (%)	Worker satisfaction (%)	Customer satisfaction (%)
Artificial group	96.38	95.67	97.55
Intelligent positioning group	74.27	76.32	63.57
*t*	3.687	4.267	2.517
*P*	0.015	0.011	0.009

## Data Availability

The data underlying the results presented in the study are available within the article.
